RETRACTED

# Inspecting Decorative Ceramic Defects by Fusing Convolutional Neural Network and Image Recognition

**DOI:** 10.1155/2022/3983919

**Published:** 2022-08-21

**Authors:** Kaiyan Jin, Chunbin Wang

**Affiliations:** ^1^Jingdezhen Ceramic University, Jingdezhen 333403, Jiangxi, China; ^2^Huzhou University, Huzhou 313000, Zhejiang, China

## Abstract

The intelligent inspection of ceramic decorative defects is one of the hot research at present. This work aims to improve the defect inspection automation of finished decorative ceramic workpieces. First, it introduces the multi-target detection algorithm and compares the performance of different network models on the public data set. Second, the initial images are collected on the spot. The initial pictures are easy to produce noise in actual deployment, affecting the image quality. Therefore, image preprocessing is performed for the initial images, and a median filtering method is used to calculate the denoising. Finally, the original You Only Look Once version 3 network model is realized. Based on this, the decorative ceramic-oriented Automated Surface Defect Inspection model is proposed. Then, decorative ceramic defect images are inputted for model training. The experimental conclusions are deeply studied and analyzed. The results show that the proposed decorative ceramic-oriented Automated Surface Defect Inspection model based on Deep Learning technology has good feature extraction and inspection ability. The detection accuracy is 94.90% on the test set, and the detection speed reaches 25 frames per second. Compared with the traditional manual inspection method, the proposed model greatly improves the inspection effect and can meet the on-site inspection requirements of surface defects of decorative ceramics under complex backgrounds. It is of great significance to improve the quality inspection efficiency and economic benefits of China's decorative ceramics industry.

## 1. Introduction

The purpose is to improve ceramic decoration's Automated Surface Defect Inspection (ASDI) level. Deep Learning (DL) is the technical representative of the new generation of Artificial Intelligence (AI). First, DL is compared with Shallow Learning, which features less expression ability against complex problems and deep patterns [1]. DL is an advanced step to the traditional model. It includes more hidden layers in the computer network. It fits more complex functions, which thus plays a more prominent role in deeper and multilevel applications, especially in the fields of image processing and feature recognition [2]. In particular, in image processing and application, Convolutional Neural Network (CNN) is also the key research core in learning [3].

RETRACTED

Defect inspection is also an important link in the production process of decorative ceramics, and it is also essential to control the quality [4]. At present, the defect inspection of decorative ceramics and formed workpieces mostly depends on manual inspection, with low efficiency. The inspection results are closely related to technicians' experience, so the test results' stability cannot be guaranteed [5]. In order to improve the quality automation of decorative ceramic production lines, reduce the production cost, and increase the accuracy and speed of defect measurement, this work develops a decorative ceramic-oriented ASDI algorithm based on DL [6].

The network model selection follows the principle of improving the current decorative ceramic-oriented defect inspection and intelligence level and guaranteeing the stability of the current detection. First, this work introduces various target detection algorithms and compares and analyzes the reliability performance of these network models in real data sets. Second, a CNN is constructed. Specifically, *y*_*j*_^*l*^=*f*(∑_*i*=1_^*N*^*x*_*i*_^*l*−1^*∗ω*_*i*,*j*_+*b*_*j*_^*l*^), *j*=1,2,…, *M*, where *ω*_*i*,*j*_ represents convolution kernel. *b*_*j*_^*l*^ is the offset. *f*() denotes the activation function. *x*_*i*_^*l*−1^ indicates input. *y*_*j*_^*l*^ stands for the output feature of the convolution layer. Then, the original You Only Look Once version 3 (YOLOv3) is established to preprocess the collected images. Finally, the YOLOv3 network is trained. The experimental conclusions are deeply studied and analyzed. The test results are compared with the existing research to show the intelligence level of the proposed decorative ceramic-oriented ASDI algorithm. Intelligent ceramic defect inspection methods can improve the automatic inspection quality and save labor costs. Hence, the decorative ceramic-oriented ASDI algorithm greatly improves the decorative ceramics industry's quality inspection efficiency and economic benefits. The innovation lies in using the YOLOv3 network model for image processing and its application in ceramic defect inspection. The finding is of positive significance to the further development of Neural Networks (NNs).

## 2. Literature Review

The surface defect inspection of industrial products has always been a hot direction of industrial production and academic research. The traditional surface defect inspection method mainly uses the physical characteristics of objects, such as acoustic, optical, and electromagnetic, without damaging the workpiece. Machine Vision (MV) inspection technology is the most commonly used. Many manufacturers and scientific research institutes favor it because of its noninvasiveness, safety, efficiency, and automation advantages. MV inspection technology is based on image features. It needs to manually design feature extraction operators to extract target features in the image and then complete defect inspection through Machine Learning classifiers. Threshold segmentation and edge FE methods are commonly used [7]. Fast inspection speed is its biggest advantage. Only a small number of samples need to be trained to achieve the effect of defect inspection. However, the difficulty of this method is to design of FE operators. Different defects have distinct characteristics, so multiple FE operators must be designed according to the characteristics of each type of defect. This requires a large workload and poor universality.

RETRACTED

Developed countries, such as the United States, Japan, and Germany, as leaders in MV, have applied many mature technologies to practical production [8]. The rapid development of the foreign MV industry is due to the unremitting efforts of countless foreign researchers. Younas et al. developed a unique architecture and algorithm set to realize the ASDI of continuous casting and hot rolling billets in steel plants [9]. Nogay et al. constructed an MV-based ASDI system. They generalized it in the printing industry by combining the image morphology processing method and algorithm parallel technology [10]. Garrido et al. established an electromechanical integrated defect inspection system based on the nonplanar mirror. They successfully inspected the image's surface defect shadows of various shapes and sizes [11]. Holmes et al. employed four different algorithms: Fourier filtering, automatic median, image convolution, and one-step threshold segmentation to inspect defects of high reflection chromium-plated rings. The research compared several algorithms' inspection accuracy and speed [12].

After the 1990s, China began to study the related technology of MV [13]. The starting point is much lower than that in foreign countries. However, domestic universities and scientific research institutes have also implemented some effective solutions. Pourkaramdel et al. realized the image defect inspection of the ball grid array chip by using the point analysis method [14]. Guan et al. successively grayed out the metal surface image, analyzed the fluctuation, combined the images with the adjacent gray difference segmentation algorithm, and realized the adaptive segmentation of metal surface defects [15]. Gauder et al. proposed an unsupervised chip surface defect inspection technology based on a convolutional denoising self-encoder [16]. The network model does not need much manual annotation during training, which enhances the availability of the method.

RETRACTED

Although the domestic research on defect inspection technology based on MV started late, it has also made many achievements. China should also recognize the gap between domestic research with foreign countries, especially the United States, Japan, and Germany, despite this progress. Meanwhile, the traditional MV-based defect inspection algorithm also has some shortcomings, such as the artificial design of the feature operator and poor algorithm universality. Especially, given a wide variety of defects with complex features, the defect inspection accuracy will be greatly reduced, which is difficult to meet practical demands.

## 3. Materials and Methods

### 3.1. The Basic Structure of CNN

CNN is a typical NN in image processing, which simulates the work of neurons in the human brain. The basic unit is artificial neural. It transmits information layer by layer and is quite apt for large-scale image processing [17]. Generally, CNN includes the input, convolution, pooling, fully connected, and output layers. The input layer is mainly responsible for network input, mostly an image number matrix. The input data go through a series of algorithm calculations by the convolution layer, pooling layer, and fully connected layer until the calculation results are outputted by the output layer [18].

#### 3.1.1. Convolution Layer

The convolution layer is the main part of the CNN. The layer-to-layer connection directly reflects the basic information as hierarchical data. Each convolution layer has several convolution kernels. The number of convolution kernels has a great influence on the recognition of CNN [19]. The convolution layer is mainly used to obtain feature maps and perform convolutions. The mathematical expression of the convolution operation reads:

(1) $$\begin{array}{c} y_{j}^{l}=f\left(\overset{N}{\underset{i=1}{\sum }}x_{i}^{l-1}*\omega_{i,j}+b_{j}^{l}\right),j=1,2,\ldots ,M. \end{array}$$

In equation (1), *ω*_*i*,*j*_ represents the convolution kernel, *b*_*j*_^*l*^ refers to the bias term, *f*() is the activation function, *x*_*i*_^*l*−1^ indicates the input, *y*_*j*_^*l*^ means the output feature map of the convolution layer, and the process of the convolution operation is shown in Figure 1.

Weight sharing is also the main feature of the convolution layer. A convolution kernel with the same parameters can be used on different image areas [20]. The weight sharing reduces the network parameters and improves the speed of simulation training and deduction [21]. The convolution layer can also perform multi-convolution operation control. It scans the input feature map through several different convolution kernels. The scanning result of each convolution kernel will get a feature map. The accuracy can be improved by using multiple feature maps [22].

RETRACTED

#### 3.1.2. Pooling Layer

The pooling layer is usually placed after the convolution layer, and its main function is to reduce the length of the feature map to reduce the network parameters [23]. The pooling layer also outputs feature maps. However, these feature maps are downsized versions of the previous layer [24]. The pooling method mainly uses the filter to eliminate the useless signal in the feature map after the convolution operation. This can greatly reduce the amount of data information and complexity while retaining the important signal [25]. Therefore, the pooling method has great advantages in reducing network parameters and network computation and improving the robustness of the network system. The general expression of the pooling operation is shown in equation (2):

(2) $$\begin{array}{c} y_{j}^{l}=\text{down}\left(y_{j}^{l-1}\right). \end{array}$$

In equation (2), *l* represents the number of layers of CNN, and *y*_*j*_^*l*^ denotes the output result of the *l* − 1 layer. The network passes the feature map of the *y*_*j*_^*l*−1^ layer through the pooling function down() to obtain the output of the *l*th layer *y*_*j*_^*l*^.

The pooling method's specific implementation process mainly includes dividing the feature map into small matrices of the same size but not crossing each other and then replacing the entire small matrix with a numerical value according to different principles [26]. Although the number of feature maps does not change after pooling, its size will significantly reduce. Only the most useful information in the feature map is saved, thus increasing the robustness of CNN modeling [27]. The schematic diagram of the pooling operation is shown in Figure 2.

In a standard CNN, the pooling layer generally only performs downsampling operations without involving activation function operations [28]. However, some models also add an activation function to the pooling layer to increase the expressiveness of the network. The mathematical expression reads:

(3) $$\begin{array}{c} y_{j}^{l}=f\left(\text{down}\left(y_{j}^{l-1}\right)\right), \end{array}$$

where down() indicates the downsampling operation, *f*() shows the nonlinear activation function, and *y*_*j*_^*l*^ illustrates the output result of the pooling operation.

#### 3.1.3. Fully Connected Layer

The fully connected layer was the most common hidden layer of the network before the convolution layer was invented. All artificial neurons in one-layer form links with all neurons in the previous level. The main feature is a large amount of data and a large operation capacity; it uses many parameters and operations to sort information [29]. The mathematical expression of the fully connected layer reads:

(4) $$\begin{array}{c} y_{j}^{l}=f\left(\sum_{i=1}^{n}\omega_{ji}^{l}\cdot x_{i}^{l-1}+b_{j}^{l}\right), \end{array}$$

where *ω*_*ji*_^*l*^ means the weight, and *b*_*j*_^*l*^ denotes the bias corresponding to the weight.

RETRACTED

In the CNN, after multilevel convolution layers and pooling layers, one or more fully connected layers are connected, and the acquired higher-level features are fused. Then, the fused features are converted into a probability distribution, and the analytical conclusion of the network is provided according to the probability distribution through the output layer [30].

#### 3.1.4. Activation Function

The activation function is the main part of the CNN, and it is generally applied in the convolution layer [31]. The activation function is created by imitating the working mode of transmitting information between the neural units of the artificial brain. That is, when the activation degree of the neuron exceeds a certain threshold, the neuron will be activated. The signal of this neuron will be transmitted backward, so the working mode of the activation function is also similar [32]. Several common activation functions are described as follows:

The Sigmoid function is often used in binary classification models. It can map the input value of any interval to the (0, 1) interval. Its mathematical expression reads:

(5) $$\begin{array}{c} f\left(x\right)=\frac{1}{1+e^{-x}}. \end{array}$$

Tangent Hyperbolic (Tanh) function is a trigonometric function. Its function curve is similar to Sigmoid. The difference is that the output range of the Tanh function is (−1, 1), which is larger than the output range of the Sigmoid function. The gradient of the function near the origin is also larger. Its mathematical expression reads:

(6) $$\begin{array}{c} f\left(x\right)=\frac{e^{x}-e^{-x}}{e^{x}+e^{-x}}. \end{array}$$

Rectified Linear Unit (ReLU) can help the network model converge faster by fixing the gradient vanishing problem. It is one of CNN's most commonly used activation functions [33]. The ReLU activation function takes the maximum value in different intervals, and its mathematical expression reads:

(7) $$\begin{array}{c} f\left(x\right)=\left\{\begin{array}{c} x,\;x\geq 0,\\ 0,\;x<0. \end{array}\right. \end{array}$$

Equation (7) indicates that the ReLU function has unilateral inhibition, generating sparsity among neurons. When the input value is positive, ReLU output equals the input, and the derivative is 1. When *x* is negative, ReLU outputs 0, and the derivative is 0. The derivative of the ReLU function is easy to calculate, accelerating network convergence. The derivative of the ReLU when the input is positive is 1, ensuring that the gradient can be transmitted stably during the backpropagation process. Thereby, it eliminates the problem of vanishing gradient during CNN training.

RETRACTED

The YOLOv3 algorithm is the most representative network in the one-stage target detection model. It is also a defect testing model based on the regression idea [34]. YOLOv3 is the latest version of the Polo series proposed by Remon at the beginning of the 21st century. The focus is to overcome the insufficient accuracy of the previous two versions. YOLOv3 has seen a substantial improvement over YOLOv2 [35].

### 3.2. Image Filtering and Denoising

#### 3.2.1. Median Filtering

Median filtering is a classic nonlinear filtering algorithm. The algorithm's implementation process mainly includes selecting a template of a special specification, covering a small range of the image in turn according to certain rules. Then, the pixel points are arranged according to the number of image values within the coverage range. Finally, the median value is chosen as the image value covers the center point. Median filtering can effectively reduce the problem of sudden changes in image pixel values, especially for salt and pepper noise. For a set of data *p*_1_, *p*_2_, *p*_3_,… *p*_*n*_, sort *S*_1_, *S*_2_, *S*_3_,…, *S*_*n*_ in descending order, then the mathematical definition of the median value is shown in equations (8) and (9):

(8) $$\begin{array}{c} M=\text{Media}\left\{p_{1},p_{2},p_{3},\ldots ,p_{n}\right\}=s_{\left(n+1\right)/2}, \end{array}$$

(9) $$\begin{array}{c} M=\text{Media}\left\{p_{1},p_{2},p_{3},\ldots ,p_{n}\right\}=\frac{\left(s_{n/2}+s_{n/2+1}\right)}{2}. \end{array}$$

In equation (8), *n* of *s*_(*n*+1)/2_ is an odd number. In equation (9), *n* of (*s*_*n*/2_+*s*_*n*/2+1_)/2 is an even number.

#### 3.2.2. Mean Filtering

Mean filtering is a linear filtering algorithm. The basic principle is to use a special template to cover a small area of the image in turn according to certain rules. Then the image values in the center of the covered area are averaged. Finally, the mean is used to replace the image values in the center of the template range to obtain the purpose of denoising. The neighborhood *S* is selected for each pixel (*x*, *y*). Afterward, the mean of *S* is used as the value of the pixel (*x*, *y*). The filtering operation is performed to obtain the image *g*(*x*, *y*). Its mathematical expression is shown in equation (10):

(10) $$\begin{array}{c} g\left(x,y\right)=\frac{1}{N}\sum_{\left(x+m,\;y+n\right)\in S}f\left(x+m,y+n\right). \end{array}$$

In equation (10), *N* is the number of pixels in the neighborhood *S*. For the mean filtering algorithm, the larger the range of the neighborhood *S* is, the better the denoising effect is. However, the image may lose some detailed feature information. Therefore, choosing an appropriate size for the neighborhood *S* is necessary to balance noise suppressing and image blurring.

RETRACTED

The experiment mainly focuses on the salt and pepper noise with a high inspection accuracy. It takes small crack defects as an example. First, the original image with small crack defects is added with salt and pepper noise. Second, different filtering and denoising techniques are used, respectively. Finally, the performance of different filtering and denoising techniques are compared.  Figure 3 compares the processing results of the above algorithms.

Figure 3(a) shows the original image of small crack defects.  Figure 3(b) illustrates the result after adding salt and pepper noise to the original image.  Figure 3(c) presents the result after median filtering and denoising.  Figure 3(d) displays the resulting image after the mean filtering and denoising. Apparently, the effect of median filtering is the best, and the calculation method of the median filtering algorithm is relatively simple and takes less time.

### 3.3. Data Collection and Data Set Construction

There is no open-source and available defect inspection dataset of decorative ceramic on the Internet, so the required datasets are collected from the field. The obtained data set contains three kinds of defects: small cracks, hard cracks, and crawling. Small cracks are mainly manifested through the body and glaze layer on the decorative ceramic body, usually in the forming stage. Hard cracking is the cracking, dark cracking, or cracking with a large opening after firing, which is usually caused by the vibration of the product during transportation. Crawling occurs when the partial glaze layer of the product falls off after firing and misses to form an exposed porcelain body, which usually occurs in the firing stage. Sample images of different kinds of defects are shown in Figure 4.

Defects affect the quality of decorative ceramics. In practice, the precise definition of cracks can be tricky, so all on-site judgments rely on experienced masters. A total of 2,331 original images are collected.

### 3.4. Experimental Steps

The experimental steps of the proposed decorative ceramic-oriented ASDI algorithm are shown in Figure 5.

Here is the specific experimental flow:

1. Image preprocessing. Mean filtering is used to remove possible noise in the original image.
2. Labeling of raw data. LabelImg program is used to label the obtained raw data to obtain Extensible Markup Language (XML) documents related to the data. Then Python script is adopted to batch the standard training set of XML documents.
3. Construction of the YOLOv3 network model. The convolution, pooling, normalization, activation functions, and other functions provided by the open-source DL framework Tensorflow and Keras are used to build the YOLOv3 network model and initialize the model.
4. The data set (including images and corresponding XML files) generated in Step (2) is inputted into the network model in batches to train YOLOv3 iteratively. Here, the Adam optimizer is selected. Meanwhile, the backpropagation algorithm updates the parameters until the loss value of the network tends to stabilize, and the training is completed, saving the parameters of the final model.
5. In the network model experiment, the defect inspection set of decorative ceramic is added as an input to the YOLOv3 model after training, and the detection results are recorded for big data analysis.

RETRACTED

### 3.5. Network Training

The model training adopts the two-stage training method. In the first stage, the Adam model optimizer is used. Epoch is set to 200 rounds, the learning rate is set to 0.001, the learning rate decline parameter is not set, and the batch size is set to 16. Sixteen images are randomly selected from the training images every time to train the model. As long as the last three layers of the model are not frozen, only the last three layers will be trained, and the parameters will be updated accordingly.

The second stage follows right after the first-stage training, using the model parameters of the first stage as the initial parameters of the network. The second stage unfreezes all hidden layers to participate in model training. Adam optimizer is adopted, and batch size is set to 8. Epoch is set to 600 rounds, and the starting round is 200. This is to facilitate viewing the details of the training process in Tensorboard. The learning rate is set to 0.0001, the momentum parameter is set to 0.1, and the patience value is set to 3. When the model loss function does not decrease for three rounds, the learning rate is reduced to one-tenth of the original. The training continues until the loss function does not decrease. Additionally, the early stopping technology is also used in the training process, and the patience value is set to 10. This means that the network converges when the loss function of the YOLOv3 network exceeds ten rounds and does not decrease. Then, the network training will stop in advance. Other hyperparameters adopt default values.

## 4. Results and Discussion

### 4.1. Distribution of the Original Data

Figure 6 illuminates the proportion of various defects in the collected samples.

RETRACTED

In Figure 6, there are three kinds of ceramic surface defects. XLW is the acronym Pinyin “Xiao Lie Wen,” which means small crack, accounting for 59%. YK is the acronym Pinyin “Yuan Kong,” which means crawling, accounting for 29%. YL is the acronym Pinyin “Ying Lie,” which means hard crack, accounting for 12%.

### 4.2. Training Results of YOLOv3 Original Model

The network model stops training at the 262nd round after over ten hours, which means that the network model has converged. The loss function value drops to 7.7381 when it converges, and the learning rate drops to 1.0 × 10^−10^. The parameters of the model training process are shown in Figure 7.

Figure 7 draws the training loss function curve and the learning rate of the YOLOv3 original model. Apparently, in the first-stage training, the loss function curve stabilizes and improves after 80 epochs and stops decreasing. This is the end of first-stage training. The second-stage training is performed at the 200th epoch. It is observed that the loss function decreases significantly with the decrease in the learning rate. Meanwhile, Figure 7(b) shows that the learning rate also decreases from the 237th epoch. Then, the learning rate stabilizes at about 252 epochs, and the loss function of all network models also remains stable. Training can be ended early at the 262nd epoch because the network triggers the early stopping mechanism. Compared with the literature YOLOv3 model by Huang et al., the training effect of the YOLOv3 model reported here is better [36].

### 4.3. Test Results of the YOLOv3 Network Model

After obtaining the trained model file, a Python script can be written to test the model performance on the validation set. The experimental results of the YOLOv3 network model are shown in Figure 8.

Figure 8 represents that the original YOLOv3 model can still obtain a good result on the decorative ceramic-oriented ASDI without modifying the basic structure and initial parameters of the original YOLOv3 model. The YOLOv3 model presents a high defect inspection accuracy, thus confirming the reasonability of using the YOLOv3 algorithm as the decorative ceramic-oriented ASDI. Wan et al. observed that the YOLOv3 model had certain advantages in inspection tasks. The finding is consistent with this work's research conclusions [37].

### 4.4. Detection Results of Various Defects by the YOLOv3 Network Model

The actual experimental results are carefully observed. It finds that the proposed decorative ceramic-oriented ASDI model presents a more than 90% inspection accuracy against ceramic crack defects except for small cracks. Specifically, the defect accuracy against hard crack has the highest detection accuracy, which exceeds the Area Precision (AP) of 96.62%. The proposed decorative ceramic-oriented ASDI model's detection speed can also exceed 32 frames per second (FPS). The inspection results of three kinds of defects are shown in Figure 9.

RETRACTED

Against small cracks, the proposed decorative ceramic-oriented ASDI model presents a relatively poor detection result, with only 79.24% AP.  Figure 10 reveals a partial image with small crack defects.

Figure 10 demonstrates that the small crack defects have quite complex surface characteristics, making them extremely difficult to inspect. For example, small-crack defects in Figure 10(a) spreads wildly to thousands of pixels in the image. Small-crack defects in Figure 10(b) are less obvious and occupy less than ten pixels. Lastly, small-crack defects in Figure 10(c) are more obvious but relatively unidirectional. This complex feature is also the main factor that causes the poor measurement accuracy of the model against the small crack defects. The accuracy of the proposed ASDI model is more than 90%, except for small crack defects. Compared with the latest research by Wang et al., the accuracy of the proposed decorative ceramic-oriented ASDI model is higher. Thus, the proposed decorative ceramic-oriented ASDI model has certain advantages and novelty [38].

## 5. Discussion

This work confirms the superiority of the YOLOv3 model in detection. The application of the YOLOv3 model in ceramic defect inspection shows that the inspection accuracy of hard crack and shrinkage round holes is more than 90%. The inspection accuracy of small cracks is low, 79.24%. Presumably, small cracks are generally complex, and the defects are not obvious, which has higher requirements for the detection model [39]. The inspection accuracy of Xia et al. research on small cracks in ceramic defects is higher than in this work. Hence, there is still much room for improvement in this work [40]. Compared with the current automation level of ceramic defect inspection in Chen et al., the results of this work have been improved [41]. By adding DL, the intellectualization of ceramic defect inspection technology has been improved.

## 6. Conclusion

First, this work expounds on the structure and characteristics, multifeature image fusion, the basic principle of image noise reduction, and the loss function design of the YOLOv3 network. Second, network training parameters are set, and the experimental environment is configured. Finally, evaluation experiments are designed to test the performance of the proposed decorative ceramic-oriented ASDI model based on YOLOv3. The finding implies that the proposed decorative ceramic-oriented ASDI model based on YOLOv3 can obtain better measurement results on the defect dataset of decorative ceramics. Therefore, YOLOv3 is suitable for defect inspection of decorative ceramics. However, due to the relatively low measurement accuracy of small cracks, the quality of the overall model still has room for improvement. For the actual production, higher measurement accuracy is required. Therefore, future work is expected to improve the proposed decorative ceramic-oriented ASDI model based on YOLOv3 in its overall accuracy. The aim is to expand the application of DL technology in decorative ceramic defect inspection.

RETRACTED

## Figures and Tables

**Figure 1:** The process of the convolution.

**Figure 2:** Schematic diagram of max pooling and average pooling operations.

**Figure 3:** Results of different filtering algorithms for small crack defects. (a) Original image. (b) Add salt and pepper noise. (c) Median filtering. (d) Mean filtering.

**Figure 4:** Schematic diagram of various defects. (a) Small cracks. (b) Hard cracking. (c) Crawling.

**Figure 5:** Experimental flowchart.

**Figure 6:** Distribution of the original data.

**Figure 7:** The parameters of the model training process. (a) Loss. (b) Learning rate.

**Figure 8:** The experimental results of the YOLOv3 network model.

**Figure 9:** Detection results of various types of defects. (a) Small cracks. (b) Hard crack. (c) Crawling.

**Figure 10:** Small crack defects of different types. (a) The first type of small cracks. (b) The second type of small cracks. (c) The third type of small cracks.

## Data Availability

The data used to support the findings of this study are available from the corresponding author upon request.
